# Lung Cancer Stage Prediction Using Multi-Omics Data

**DOI:** 10.1155/2022/2279044

**Published:** 2022-07-16

**Authors:** Wei Li, Binchun Liu, Weiqian Wang, Can Sun, Jianpeng Che, Xuelian Yuan, Chunbo Zhai

**Affiliations:** ^1^Second Ward, Department of Thoracic Surgery, Weifang People's Hospital, Weifang 261041, China; ^2^Qingdao Geneis Institute of Big Data Mining and Precision Medicine, Qingdao 266000, China; ^3^Geneis (Beijing) Co., Ltd., Beijing 100102, China

## Abstract

Lung cancer is one of the leading causes of cancer death. Patients with early-stage lung cancer can be treated by surgery, while patients in the middle and late stages need chemotherapy or radiotherapy. Therefore, accurate staging of lung cancer is crucial for doctors to formulate accurate treatment plans for patients. In this paper, the random forest algorithm is used as the lung cancer stage prediction model, and the accuracy of lung cancer stage prediction is discussed in the microbiome, transcriptome, microbe, and transcriptome fusion groups, and the accuracy of the model is measured by indicators such as ACC, recall, and precision. The results showed that the prediction accuracy of microbial combinatorial transcriptome fusion analysis was the highest, reaching 0.809. The study reveals the role of multimodal data and fusion algorithm in accurately diagnosing lung cancer stage, which could aid doctors in clinics.

## 1. Introduction

In most cases, cancer is considered a genetic disease of unknown cause, a problem that humans have not yet overcome. In recent years, the morbidity and mortality of cancer have been increasing rapidly worldwide, and it is the main cause of death for many human beings. Among them, lung cancer accounts for 11.6% of the total cancer incidence and 18.4% of the total cancer mortality [1–3]. In the United States and East Asia, lung cancer is the main killer of cancer [4, 5]. Worldwide, more than 1 million people die of lung cancer every year [6–8]. Lung cancer is a common primary lung tumor. It is a complex disease caused by the interaction of multiple genes and multiple pathways, which can spread around or even throughout the body. Staging is a method of classifying the severity and extent of a tumor's spread according to its growth and development. The staging of lung cancer can be aggregated into stage I, stage II, stage III, and stage IV. Among them, stage I is the earliest stage, and stages II, III, and IV are the middle and late stages. The key to the treatment and prognosis of lung cancer is staging [9, 10]. Accurate staging can provide strong support for doctors to formulate accurate treatment plans for patients and improve the survival rate of patients [11]. Surgical resection is the first choice for patients with early-stage lung cancer, while patients with advanced stage can receive corresponding preoperative induction chemotherapy according to the stage of cancer to improve the survival period of patients [12]. Therefore, staging of lung cancer is of great significance to the management and treatment of patients. It can not only effectively judge and evaluate the survival cycle of patients, but also provide effective guidance and strong support for doctors to formulate appropriate treatment plans for patients. Chest CT and MRI are traditionally important means for doctors to judge the stage, but because imaging often underestimates the stage of cancer, about 55% of patients have inaccurate staging results [13]. Computed tomography is an important method for clinical diagnosis and staging and has a high sensitivity for the diagnosis of malignant lesions [13–17], but unfortunately, only advanced malignant cells can be detected, resulting in a low patient survival rate [18]. It is imperative to find other means of staging, diagnosis, and prediction.

Studies have found that the occurrence of lung cancer is related to genetic factors. With the development of molecular biology and the advent of the era of big data, machine learning has been widely used in the staging and classification of cancer [19–22]. Researchers have analyzed the impact of gene expression on the occurrence and development of cancer from the perspective of genomics [23–25]. For example, miRNA biomarkers based on gene expression can classify samples from gastritis to gastric cancer at different stages of development [26]. At present, DNA microarrays have been widely used in cancer research, providing accurate classification information and prediction information for tumor staging, patient survival rate, and other states and providing direction for precision medicine [27]. Lung cancer is a gene-related disease that causes dramatic changes in gene expression in tumor cells. Staging and prediction of lung cancer using genes retained in tissues can further enhance the understanding of the pathogenesis of cancer and the process of development and metastasis. At present, the research on lung cancer and genes has a large number of results. For example, in early-stage non-small cell lung cancer (NSCLC), the gene expression level of gene Bmi-1 showed a regularity of increasing first and then decreasing [28]. In addition, the gene BRCA2 mutation will greatly increase the risk of lung cancer. Studies have shown that the risk of lung cancer in smokers with BRCA2 mutations is twice that of the general population [29]. Mutations in the gene EGFR accelerate the abnormal growth and division of cells, leading to the development of tumors. In advanced lung cancer, there is a high EGFR mutation rate [30]. However, as studies have found that the predictive power of gene expression profiles is poorly understood compared to clinical and pathological predictions, the use of a single type of signature may not be sufficient for accurate lung cancer staging.

It is well known that human health is closely related to the microbiome, which has emerged as a key regulator of carcinogenesis and cancer cell immune responses. The human microbiota is an ecological community of symbiotic and pathogenic microorganisms. Although most microorganisms are symbiotic, in some cases, microorganisms that are beneficial or harmless to the human body can promote the occurrence and development of cancer [31–33]. The microbiome may promote the occurrence and development of cancer through various pathways such as inflammatory, immune dysregulation, and product metabolism [34]. Studies have found that the microbiome is closely related to the occurrence and development of lung cancer. The lung commensal microbiota reduces lung inflammation and regulates immune tolerance through the recruitment of dendritic cells (DC), T regulatory cells, and other cells. Dysregulation of the lung microbiome may induce immune dysregulation to induce cancer development [34]. As studies have shown, there is a significant relationship between *Mycobacterium tuberculosis* (TB) and lung cancer [35]. *Ruminococcus*, *Eubacterium*, and *Bifidobacterium adolescentis* were enriched in lung cancer patients. Gut microbes can affect the immune function of the lungs through different mechanisms. The gut microbiota is closely related to the permeability of the gut and respiratory tract. Intestinal microbial dysbiosis may increase the permeability of the gut, allowing antigens to invade the bloodstream and the whole body, thereby promoting a systemic inflammatory immune response and affecting lung function. In addition, there may be differences in the composition and abundance of microorganisms in cancer samples at different stages [36]. Microorganisms can be used to predict tumor staging and further improve patient survival. For example, *Enterococcus haiii* and *Barnesella enterica* were significantly expressed in advanced lung cancer. At present, the research on microorganisms and lung cancer is still in the preliminary stage, and there are more contents waiting for us to study.

This paper uses multi-omics to jointly study lung cancer staging and prediction, reduce the instability of gene prediction, further explore the abundance of microbiome in lung cancer staging, and use multitype features to further improve the accuracy of staging prediction.

## 2. Materials and Methods

### 2.1. Data Preprocessing

Clinical data of 189 lung cancer patients were downloaded from TCGA (https://dcc.icgc.org/releases/release_26/), and microbial data of 1524 cases were obtained from the nature article “Microbiome analyses of blood and tissues suggesting a cancer diagnostic approach.” To obtain complete genomic information, whole genome sequencing (WGS) samples in tissue samples were selected, resulting in 189 samples (see Table 1 for details).

### 2.2. Gene Expression Profiling

In living organisms, under the influence of different factors such as time, environment, and developmental degree, gene expression changes all time. During the occurrence and development of tumors, many genes that are usually silenced begin to be highly expressed, and the expression of those normally expressed genes may be downregulated. It is precisely these genes whose expression changes from normal gene expression that their presence initiates the occurrence of tumors. Therefore, it is essential to study these differentially expressed genes if we want to study the mechanism of tumorigenesis [26] and drug response [37, 38]. The DESqe2 package in R can be used for expression analysis. DESeq2 is a method based on the negative binomial distribution, which uses local regression to infer mean and variance, and uses dispersion and fold-change shrinkage estimates to improve stability [35, 39, 40]. The standardization principle of DESeq2 is to improve the status of moderately expressed genes, which can well control false positive errors and have high sensitivity and specificity [41]. The DESeq2 analysis of differentially expressed genes is roughly divided into three steps: The first step is preparing data and forming a gene expression matrix; the second step is calculating the differential fold list to obtain the differential fold change and significant *P* value of each gene, define thresholds to screen for differentially expressed genes, and distinguish upregulated and downregulated genes by “up” and “down.” The threshold for screening differentially expressed genes is set as: p.adj < 0.05&abs(log2FoldChange) > 1.

### 2.3. Enrichment Analysis

Enrichment analysis is a way to understand the functional propensity of a gene set and is widely used in the field of omics research. Common enrichment analysis methods include GO enrichment analysis and KEGG enrichment analysis. GO (gene ontology) is a database established by the Gene Ontology Consortium to describe the function of gene products. GO enrichment analysis is mainly used for the enrichment degree of differential genes with GO terms: the darker the color, the more significant [42]. KEGG is a database established in 1995 that integrates genomic, chemical, and systematic functionalities and can be used to predict protein interaction networks of various cellular processes. KEGG pathway enrichment analysis is often applied to the functional annotation of differentially expressed genes to understand the related functions and pathways of differentially expressed genes [43].

### 2.4. Microbial Analysis

Microorganisms are ubiquitous and play an important role in the biological functions of the human body [44–46]. Studies have shown that the specific composition of the microbiome is associated with a variety of diseases, such as *Citrobacter rotavirus* infection can promote the development of colon cancer [47]. Microbial genome research can deepen the understanding of the pathogenic mechanisms, important metabolism, and regulatory mechanisms of microorganisms by utilizing the important functional genes of microorganisms through complete genomic information. Different microorganisms play different roles [48]. Determining the abundance of some key populations is therefore important for understanding the role of microbial communities. The Wilcoxon rank sum test (Mann–Whitney test) was used to perform differential analysis of relative abundances.

### 2.5. Model Building and Feature Selection

With the advent of the era of big data, machine learning has been widely used in cancer classification and prediction research. Machine learning algorithms can be roughly divided into three categories: supervised learning, semi-supervised learning, and unsupervised learning [49–55]. Random forest is a supervised learning model [56, 57], and the basic unit is a decision tree [58]. A random forest consists of many decision trees, each node of the decision tree is a condition of a single feature, and there is no connection between these decision trees. The general steps of random forest classification are as follows: First, m training sets are randomly generated, each training set is a set of samples, and each training set is used to construct a decision tree; secondly, N optimal features are used to build a tree, and each leaf node represents the type of the last judgment. Not every feature can be selected when the decision tree is divided into nodes. When dividing each node, K features are randomly selected, and the optimal n features are selected from the k features for dividing nodes; finally, a large number of decision trees form a forest. The predicted staging type is the largest vote in the decision tree.

The index used for division in this paper is the Gini index. The smaller the Gini index, the better the feature. The importance score of each feature can be calculated and ranked by the Gini index. The calculation process is as follows.

*G* stands for Gini index, *S* stands for importance score, *F* = {f_1_, *f*_2_, ⋯, *f*_*n*_} stands for feature, *C* stands for staging type, and ∣*C*∣ stands for the number of types. The importance score of each feature is the sum of the importance scores of each feature on each tree and the normalized value. The formula for calculating the Gini index is

(1) $$\begin{array}{c} G=1‐\overset{\left|\text{C}\right|}{\underset{\text{c}=1}{\sum }}{\text{p}}_{\text{mk}}^{2}. \end{array}$$

Among them, *c* represents the stage category, which *p*_*mk*_ represents the proportion of category k in node *m*.

Assuming there are *t* trees, the importance scores of *f*_*i*_ features are

(2) $$\begin{array}{c} S_{i}^{*}=\overset{t}{\underset{j=1}{\sum }}\underset{m\in M}{\sum }\left(G-G1-G2\right). \end{array}$$

Among them, *G*1 and *G*2 represent the Gini index values of the two new nodes before and after the branch, respectively.

Then, the formula for calculating the importance score of the *f*_*i*_ feature is

(3) $$\begin{array}{c} S_{i}=\frac{S_{i}^{*}}{\sum_{j=1}^{t}S_{j}}. \end{array}$$

Select the top n features with the highest scores to participate in the next step of classification.

## 3. Results

### 3.1. MRNA Differential Expression Analysis

Use Deseq2 in R language to perform differential analysis on mRNA data to select differential genes. The results are visualized, and the resulting volcano map is shown in Figure 1(a). Among these genes, there were 291 differentially upregulated genes and 128 differentially downregulated genes. Among them, REG4, CALCA, PHOX2B, and other genes were significantly downregulated, and FOXI1, CYP1A1, LGI1, DLK1, and other genes were significantly upregulated.

To more intuitively present the relationship between the global variation of differentially expressed genes and the expression of multiple genes, the following heat map was drawn. Due to the large number of differentially expressed genes and samples, the top 10 genes of the up- and downregulated genes and twenty random samples were selected to draw a heat map. The detailed results are shown in Figure 1(b). The graph of Figure 1(b) shows that the expression of these 20 genes is different in the early stage and the middle and late stage of lung cancer. Each small fragment represents a gene, the color of the fragment represents the level of gene expression; the darker the color, the higher the expression level (red represents gene upregulation, and blue represents gene downregulation). The segments on the bottom represent different lung cancer stages, and the vertical lines on the right represent different genes.

To gain a deeper understanding of the functions of the differential genes, GO enrichment analysis and KEGG analysis were performed on the differential genes. The level of significance was set at *p* value 0.05. In this paper, the top 10 pathways with the smallest *p* value were selected for display. The detailed results are shown in Figures 1(c) and 1(d).

The enrichment results showed that these genes were significantly enriched within cellular metabolism, especially digestive metabolism. In addition, some genes are also enriched in axonal dynein complex assembly and carbohydrate transport. All biological activities require energy, and digestion provides cellular energy for all cellular activities. In addition, genes were enriched through the cAMP signaling pathway (cAMP). The cAMP signaling pathway is a type of cyclic nucleotide system whose levels are regulated by adenylate cyclase (AC). cAMP controls a variety of cellular processes and plays an important role in the cellular response to many extracellular stimuli. PKA is the major cellular effector of cAMP. Upregulation of cAMP levels inactivates GSK3ALPha and GSK3Beta through a PKA-dependent mechanism, thereby promoting neuronal cell survival and preventing tumorigenesis.

### 3.2. Microbial Difference Analysis

There is a large microbial community in the human body, and relative abundance analysis of key microbial populations can help to enhance our understanding of microorganisms. In this paper, the relative abundance difference analyses of 1524 genera were performed using the Wilcoxon rank sum test. The screening condition was set as *p* < 0.05, and finally 87 differential genera were obtained. The significant condition *p* < 0.01 was set, and 8 different genera were obtained. The detailed results are shown in Figure 2.

The relative abundances of *Ureaplasma*, *Kutzneria*, and *Hungatella* in the early stage of lung cancer were higher than those in the middle and late stages, and the relative abundances of *Lentimicrobium* and *Alloaction synnema* in the middle and late stages were higher. *Ureaplasma* is the most common *Mycoplasma genitalium* isolated from the male and female genitourinary tracts and is the most common potential pathogen. Studies have shown that *Ureaplasma* can cause non-gonococcal urethritis in men [59]. In addition, the metabolites of vitamin D, 25-OH-D and 1*α*,25-(OH)2-D, play an important role in the control of cell proliferation and differentiation, gene transcription, and other processes and can inhibit the proliferation of cancer cells. Compared with traditional methods, the conversion of vitamin D to 25-OH−D and 1*α*,25-(OH)2−D by microorganisms is more promising. *Kutzneria* has great potential to generate metabolites 25-OH−D and 1*α*,25-(OH)2−D.

### 3.3. Gene Expression Profiles Perform Better at Predicting Lung Cancer Stage

This paper used a random forest classifier model to predict the stage of patients. Take 70% of the dataset as the training set and 30% of the dataset as the test set. The test set does not participate in the training of the model. Here, the prediction results of the random forest model on the microbial dataset, the mRNA dataset, and the microbial + mRNA dataset are discussed separately, and the prediction results after feature fusion are discussed. This paper uses AUC, recall, precision, and ACC to evaluate the results of the model.

On the microbial dataset, the Wilcoxon rank sum test was used to select the top 1000 most abundant features. Use 5-fold cross-validation random forest to select features. After many trials, when the number of features reaches 90, the value of AUC remains stable. Use random forest to filter the 90 features with the highest importance score in each sample to form M ∗N input matrix, where M is the number of samples and n is the number of features. It is used as the input matrix for the next classification prediction. After training, the predicted AUC of the microorganism test dataset is 0.715. ACC, recall, and precision were 0.702, 0.741, and 0.667, respectively. On the mRNA dataset, the random forest of 5-fold cross-validation is used to select features. After many experiments, the 160 genes are characterized. Through the random forest classifier model test, the classification prediction AUC is 0.749. ACC, recall, and precision were 0.719, 0.778, and 0.667, respectively. On the microorganism + mRNA dataset, to prevent information loss, combined with the content of the previous work, the two features were fused to obtain 250 features. The AUC of classification prediction obtained by the random forest classifier model test is 0.752. ACC, recall, and precision were 0.702, 0.630, and 0.708, respectively. In addition, the 5-fold cross-validation random forest is used to select the merged features again, and the 50 features with the highest scores are obtained. After testing, the AUC of classification prediction is 0.809. ACC, recall, and precision were 0.772, 0.667, and 0.818, respectively. The detailed results are shown in Figure 3.

## 4. Discussion

In this paper, differentially expressed genes and differentially expressed microbial genera in lung cancer were studied, and the performance of multi-omics fusion in lung cancer staging prediction was studied using random forest algorithm. Insufficient, it can better improve the staging prediction ability of lung cancer.

In Figure 1, REG4, CALCA, and PHOX2B genes were significantly downregulated, and FOXI1, CYP1A1, LGI1, and DLK1 genes were significantly upregulated, and they were differentially expressed in lung cancer cells. REG4 is highly expressed in gastrointestinal tumors, colorectal cancer, pancreatic cancer, and other malignant tumors. If REG4 interacts with CD44, REG4 activation induces the proteolytic cleavage of CD44 to release CD44 intracytoplasmic domain CD44ICD, which in turn promotes the proliferation and clonal potential of cancer cells through the REG4-CD44-secretase-CD44ICD pathway [60]. Furthermore, studies have shown that REG4 expression is associated with larger tumors [61]. CALCA encodes the hormones calcitonin, calcitonin gene-related peptide (CGRP), and cataractin through alternative RNA splicing of transcripts and cleavage of inactive precursor proteins. Among them, CGRP is often expressed in the central and peripheral nervous systems and is involved in peripheral vasodilation, pain perception, gastrointestinal motility, neurogenic inflammation, and other physiological activities. The PHOX2B gene provides the command to make a protein that is active in the neural crest and is essential for the development of the autonomic nervous system. The autonomic nervous system controls bodily functions such as breathing and heart rate. In addition, PHOX2B mutations cause congenital central hypoventilation syndrome (CCHS) in humans, which is closely related to lung function [62]. FOXI1 belongs to the forkhead transcription gene family, the function of which has not been determined. The FOXI1 gene plays an important role in embryogenesis, and the protein it encodes is necessary for transcription in the kidney. Currently, more than 100 forkhead transcription genes have been identified. These transcribed genes are involved in a wide range of biological functions, including cell specification, cell proliferation, gene regulation in differentiated tissues, and tumorigenesis [63]. In addition, FOXI1 is an essential factor in pulmonary mucociliary formation, which may form mucus plugs or impair microbial clearance when lung mucociliary clearance is defective. CYP1A1 is mainly distributed in the skin, lung, gastrointestinal tract, lymphoid tissue, etc., and is related to the occurrence of many diseases, such as CYP1A1, and is related to the genetic susceptibility of small cell lung cancer. CYP1A1 Exon7 mutation is a suspected susceptibility factor for lung cancer, and it has a synergistic effect with smoking on lung cancer susceptibility [64]. LGI1, known as a leucine-rich glioma-inactivating gene, has been implicated in cancer cell motility and apoptosis. LGI1 is an invasion-suppressing gene, and reexpression of LGI1-deficient glial cancer cells results in significantly reduced cell viability and invasiveness. DLK1 is an important regulator of cell differentiation [65, 66] and is highly expressed in some tumors with neuroendocrine properties (neuroblastoma, small cell lung cancer, etc.) and plays an essential role in the occurrence and development of tumors [67, 68]. DLK1 may be an important factor in the Notch pathway. In lung cancer, cells transfected with Notch1 will activate the signaling pathway raf/MEK/MAPK, which is responsible for cell growth and neuroendocrine cell differentiation, so the cell cycle of Notch1-transfected small cell lung cancers is arrested, and tumor cells change [69, 70].

The microbial community in the human body coexists with humans, and the number of microorganisms living inside and outside the human body far exceeds the number of human cells [71]. These microorganisms provide benefit or disease susceptibility to humans through a variety of pathways. Dysregulation of the microbiota may play an important carcinogenic role at multiple levels. Microbes are closely related to various inflammatory lung diseases. In Figure 2, the abundance of *Ureaplasma* in the early stage of lung cancer is higher than that in the middle and late stage. *Ureaplasma* is associated with chronic lung disease in neonates. It has been speculated that *Ureaplasma* colonization may predispose the fetus to chronic lung disease (CLD) [72]. The urease activity of *Ureaplasma* produces ammonia through the cleavage of urea, which is associated with chronic lung disease in adults exposed to ammonia [73]. In addition, studies have confirmed that most of the clinically isolated *Ureaplasma* form biofilms in vitro and these biofilms may contribute to persistent and chronic inflammation in the body [74]. Lung cancer can be caused by a variety of factors, including bacteria, chronic inflammation, and chemical carcinogens. Few microbes directly cause cancer, but many are involved in the occurrence and development of cancer. Microorganisms generally act through the host's immune system. The highest concentration of commensal microbes in the human body is in the gut. The gut microbiota has broad effects on host immune function at steady state and during tumorigenesis and can influence local and distant tumors by affecting its immune milieu, myeloid and lymphocyte influx, and inflammatory and metabolic patterns. *Hungatella* is an anaerobic bacterium that is present in the human gut microbiota [75]. Although *Hungatella* is considered a nonpathogenic component of the gut microbiota, it has also been reported that *Hungatella* can cause sepsis in humans [76]. In addition, *Hungatella* plays a key role in the occurrence and development of intracranial aneurysms, and the reduction of *Hungatella* can lead to a decrease in the level of taurine in the blood, which may lead to the development of unruptured intracranial aneurysms. Furthermore, recent studies have shown that high abundance of *Hungatella* is significantly associated with COVID-19 [77].

Multi-omics association studies are the combination of multiple high-throughput detection research strategies applied to the common elaboration of the same scientific question. The formation of cancer is influenced by many factors. For a variety of data, it contains a variety of information. For these data, in addition to screening the microbial marker information in each group of samples through differential statistical analysis, it is also necessary to correlate the data obtained by other means (mRNA is used in this article) with the massive data of microorganisms, to obtain information related to various types of microorganisms. Change indicators associated with specific microbial species and genes. By combining the association analysis of the microbiome and the transcriptome, this paper comprehensively screened relevant features at the microbial species and host transcriptome levels to obtain more comprehensive information and further improve the accuracy of staging prediction. Multi-omics association studies can combine information at multiple levels, integrate information, and improve the accuracy of staging prediction. In the future, multiple omics can be combined for further research and application. With the development of technology, future precision medicine may be based on new diagnosis and treatment technologies, which can observe the changes of the microbiome in patients in more detail use these changes as markers of treatment and adjust the dysbiosis of the microbiome through external intervention, thereby intervening in the occurrence and development of tumors. Most microorganisms do not directly lead to the occurrence of cancer, but play a role in the regulation of the host's metabolism, immunity, and nervous system. For example, the microorganisms in the gut mainly come into close contact with the host through small-molecule metabolites. Therefore, it is possible to combine lung metabolomics and microbiome to conduct further research on lung cancer staging; analyze the interaction between the physiological role of the microbiota and its metabolites and metabolite functions, and the metabolic regulation pathways involved in microorganisms, etc.; and further explore the mechanism of microbiome interaction between hosts.

## 5. Conclusion

In this study, we performed a multi-omics association analysis of lung cancer staging by combining the microbiome and transcriptome. A random forest algorithm was used as a classification model for predicting patient stage. The classification prediction accuracy of random forest algorithm on the microbiome, transcriptome, and the combination of microbiome and transcriptome was discussed, respectively. The study found that the fusion of two omics can make up for the lack of single omics information and can improve the prediction ability of lung cancer staging, and the prediction accuracy rate is 0.752. In addition, feature screening was continued for the postfusion features, which further improved the accuracy of staging prediction of lung cancer, and the final accuracy of staging prediction was 0.809.

## Figures and Tables

**Figure 1:** (a) Volcano map. The figure compares the transcriptomes of 189 lung cancer patients. Among them, each point represents a gene, the abscissa is the fold difference, and the ordinate is the inverse of the logarithm of the *p* value. Colors are used to distinguish whether genes are differentially expressed, blue represents genes downregulated, red represents genes upregulated, and gray represents genes that are not differentially expressed. Genes with greater differential expression are farther away and are generally distributed at the endpoints of the graph. (b) Heat map. Heat map of the top 20 genes up and down, where the rows represent the stage of lung cancer and the columns represent the genes. (c)–(d) GO enrichment analysis and KEGG enrichment analysis. The horizontal axis represents the number of genes, the vertical axis represents the biological process and cell function, and the color represents the *p* value. The darker the color, the less significant the *p* value. In this paper, the top 10 pathways with the smallest *p* value were selected for display.

**Figure 2:** Boxplot and bee colony plot of the expression levels of 8 genera in different stages of lung cancer with rank sum test, *p* < 0.01.

**Figure 3:** Display of four outcome staging prediction results. (a) AUC value of staging prediction results. (b) Visual comparison chart of AUC, ACC, recall, and precision of staging prediction.

**Table 1:** Details of 189 samples downloaded from TCGA.

Cancer	Group	Number
Lung	Stage I	98
	Stages II, III, and IV	91

## Data Availability

The TCGA data used to support the findings of this study are included within the supplementary information file(s). I uploaded the file to Github due to the large amount of data (https://github.com/lx13778188130/lung-cancer-stage-prediction-using-multi.git).
